# Design of Resources Allocation in 6G Cybertwin Technology Using the Fuzzy Neuro Model in Healthcare Systems

**DOI:** 10.1155/2022/5691203

**Published:** 2022-01-10

**Authors:** Salman Ali Syed, K. Sheela Sobana Rani, Gouse Baig Mohammad, G. Anil kumar, Krishna Keerthi Chennam, R. Jaikumar, Yuvaraj Natarajan, K. Srihari, U. Barakkath Nisha, Venkatesa Prabhu Sundramurthy

**Affiliations:** ^1^Department of Computer Science, College of Science and Arts, Jouf University, Tabarjal, Al Jouf Province, Saudi Arabia; ^2^Electrical and Electronics Engineering, Sri Ramakrishna Institute of Technology, Coimbatore, India; ^3^Department of Computer Science and Engineering, Vardhaman College of Engineering, Hyderabad, India; ^4^Computer Science and Engineering, Scient Institute of Technology, Hyderabad, India; ^5^G. Narayanamma Institute of Technology and Science, Hyderabad, India; ^6^Department of Electronics and Communication Engineering, KGiSL Institute of Technology, Coimbatore, Tamil Nadu, India; ^7^ICT Academy, Chennai, Tamil Nadu, India; ^8^Department of Computer Science and Engineering, SNS College of Technology, Coimbatore, Tamil Nadu, India; ^9^Department of Information Technology, Sri Krishna College of Engineering and Technology, Coimbatore, Tamil Nadu, India; ^10^Department of Chemical Engineering, Addis Ababa Science and Technology University, Addis Ababa, Ethiopia

## Abstract

In 6G edge communication networks, the machine learning models play a major role in enabling intelligent decision-making in case of optimal resource allocation in case of the healthcare system. However, it causes a bottleneck, in the form of sophisticated memory calculations, between the hidden layers and the cost of communication between the edge devices/edge nodes and the cloud centres, while transmitting the data from the healthcare management system to the cloud centre via edge nodes. In order to reduce these hurdles, it is important to share workloads to further eliminate the problems related to complicated memory calculations and transmission costs. The effort aims mainly to reduce storage costs and cloud computing associated with neural networks as the complexity of the computations increases with increasing numbers of hidden layers. This study modifies federated teaching to function with distributed assignment resource settings as a distributed deep learning model. It improves the capacity to learn from the data and assigns an ideal workload depending on the limited available resources, slow network connection, and more edge devices. Current network status can be sent to the cloud centre by the edge devices and edge nodes autonomously using cybertwin, meaning that local data are often updated to calculate global data. The simulation shows how effective resource management and allocation is better than standard approaches. It is seen from the results that the proposed method achieves higher resource utilization and success rate than existing methods. Index Terms are fuzzy, healthcare, bioinformatics, 6G wireless communication, cybertwin, machine learning, neural network, and edge.

## 1. Introduction

Since the development of edge computing [1], it has emerged as a key strategic approach in a variety of application areas, especially in the fields of data aggregation, network connectivity, and other industrial tasks. The edge is regarded as an open platform for storage and computing applications because it is situated near a data source or an object on the network side. Edge computing is placed between the cloud and end devices and uses a high-speed data communication channel with a local data processing capability between them to transfer data with processing power equivalent to that of the cloud [2].

There are some basic facilities in the current healthcare system, but time and space are the main obstacles. Because of the existing circumstances, this is unavoidable; nevertheless, in the near future, it will not be a hindrance to progress. It is also worth noting that an ambulance service is nothing more than a vehicle for transporting patients with oxygen and road traffic priority. In addition, the current state of aged care is woefully inadequate. There is a great deal of emphasis on medical staff in the care of the older population. However, it has not been made available yet. In ambulances, most patients die on the way to or from the hospital or even before the ambulance gets there. Current healthcare systems also lack an accident detection system [3].

Real-time accident detection is needed to ensure that medical services are available immediately and on the scene. Furthermore, outbreaks like COVID-19 cannot be handled due to a lack of technological infrastructure. This includes epidemics and pandemics. In the future, a virus identical to this one is likely to surface. As a result, creating an intelligent healthcare system is critical. The high data throughput and low delay needs of 6G technology for future healthcare necessitate the use of this technology. Telesurgery, in particular, necessitates instantaneous communication. Intelligent healthcare systems will also benefit from holographic communication and augmented or virtual reality. As a result, intelligent healthcare cannot make use of 5G and 5G B5G. In the 5G era, intelligent healthcare will be largely adopted, which will propel a significant amount of progress [4].

The virtual cyberspace in the edge cloud is where the virtual representation of the end (humans and things) resides, making it a critical part of the cybertwin communication model. Cybertwin can meet three distinct needs by supplying 3 different features: network communications assistant feature, network behaviour logger feature, and digital asset feature [5, 6]. It is crucial that an end device connect to the server offering the services. The cybertwin will access the network in order to provide the required service to the end, and once that service is completed, will return the service to the end. This is the most fundamental function of the cybertwin's communications assistant. Cybertwin can be thought of as the digital representation of the goals, which allows the system to collect and log all the data about the network behaviour of the user's system. After removing sensitive information, cybertwin converts the behaviour data of the users into a digital asset for sale [7].

Cybertwin on the boundary has been configured to meet the needs of various industries, such as rapid connection and strong security. Data are being gathered at the cloud centre, while, on the other hand, edge computing features device-based processing. As end-user resources get closer to users, latency between the cloud data centre and devices decreases. This, in turn, allows for slightly improved quality of service (QoS). Also, as the number of devices that will be able to connect to the internet increases, the network bandwidth or capacity will be a major constraint on cloud computing. Likewise, the complexity of end-user requirements raises the difficulty of service allocation. Above all, excellent resource selection is critical to meeting end-user needs [8–14].

During the onset of large-scale distributed neural network use, the limited computing resources found at the edge devices present several challenges. A shortage of resources limits storage. These limitations are the shortage of energy and defects in architecture. Despite their complementary relationship and the reduced latency that they enjoy, the edge did not have the necessary resources to make use of cloud computing. A significant influence on application performance, task scheduling, and end-user QoS is the allocation or prediction of available resources. Providing an estimate of the required resources for each end-user will produce an appropriate resource plan, which should use certain parameters to estimate the amount of resources consumed. Therefore, in order to meet the user's QoS, the resource estimation needs to incorporate a task allocation strategy that is optimised for edge computing.

Historical research has identified cloud, edge nodes, and end-user devices as the requirements for neural network deployment. Neural networks are less latency-sensitive when there is increased resource allocation, but they have the potential to pass on the original source in the event of latency-critical applications. Edge users are offered distributed services via multiple hidden layers of neural networks. The neural network model predicts and then allocates energy resources in a near real-time manner, with minimal delay [7]. The distributed neural network architecture can identify when tasks get allocated to different partitions at the edge and will always use a partition with fewer resources if distributed edge nodes are utilised.

The aim is to design and implement distributed neural networks (DNNs) on edge networks with better performance, so that devices at the edge are capable of intelligent workload prediction. A long-standing constraint on computation and resourcing, represented by the trade-off between the computational load and resourcing task, has to be maintained using distributed neural networks.

Here, we developed federated learning (FL) [15, 16] as a subset of cybertwin as a preliminary model to assist with decisions related to reresource allocation. Such constraints as memory and communication complexity are incorporated into the preliminary model.

The major contribution of the proposed work is stated as follows:

- To improve the effectiveness of resource allocation decisions, the author built a FL model. With the DNN serving as a secondary model, it is now possible to use the following rules: edge resources allow zero or multiple edge devices, resources available, memory requirements, and user quality of service requirements.
- Decentralized training data distribution is a solution that optimises the reuse of valuable network resources, even in the event of an unreliable network. To distribute environments such as this, FL (each iteration) enables the edge node to compute updates to the cloud centre independent of system requirements, user cases, data size, and implementation effort.
- Conceptually, it can be said that the model compares the total number of servers connected to the data centre, the number of servers on the edge that connect to the cloud, and the response time

This study is structured as follows: Section 2 provides the network model.  Section 3 discusses the problem formulation, and Section 4 provides a detailed discussion on resource allocation using the FNN wireless healthcare model.  Section 5 evaluates the entire work with existing resource allocation models.  Section 6 concludes the entire work with possible directions for future scope.

## 2. Network Model

Edge computing fundamentals are discussed in this section, which finds it situated between the cloud and the edge devices. Storage, computation, and network services can benefit from edge computing. Edge computing has a distributed FNN wireless healthcare model that is utilised to make distributed computation possible with severely limited memory and processing power in the edge nodes and edge devices. Because edge devices are near the resources, real-time communication is possible.

The cyber twin aims to process data while providing the ability to communicate and perform computations freely. The present study uses a 3-tier architecture with an edge computing model, as shown in Figure 1.

The control BSs is responsible for data providing to the control plane that decides the required resources for the edge IoT devices. This resource allocation with uplink and downlink BSs enables user plane to allocate the resources for data communication from edge devices via edge IoT devices.

This edge device is made to generate data and make the client consume more of it. In particular, it urges clients to use more resources from the edge nodes rather than the cloud. Devices may range from smartphones to IoT sensor nodes, intelligent vehicles, and even smart cities. The edge devices collect data and communicate with each other using a sensor network. The cloud servers located in the cloud centre have significantly more energy and computing power than numerous edge devices [10].

Switches, routers, and local servers, which are typically deployed for special services, sit on the edge nodes. The compute, storage, processing, and data forwarding are all in place with these nodes. A single or multihop connection can be used to connect edge devices with edge nodes or edge servers. Computing, network, storage, and software resources are all available in the microdata centre (MDC). Cluster servers and data centres that act as storage and processing points for data received from edge devices are positioned at the top of the cloud layer.

Figure 2 shows the process of a service request when using edge computing. Users can submit requests to the administrator by using edge devices at the beginning. In order to meet the QoS user requirements, the query is stored in the edge nodes and is then passed on to the cloud centres through the edge nodes. Resources, sensor availability, service, and applications influence the statistics generated by the monitoring equipment. This equipment processes data that are sent to the edge nodes and QoS service levels for each user requirement, and these data are analysed to provide appropriate levels of service for each user. To allocate resources in an optimal manner, a FNN wireless healthcare model processes each service on an edge device locally to provide the optimal distribution of energy and bandwidth. A distributed FNN wireless healthcare model selects an existing resource and allocates it according to user QoS requirements.

## 3. Problem Formulation

The study aims to improve the allocation of energy considering all constraints for optimal consumption of energy at the IoT edge network. Furthermore, it considers various constraints including resource allocation constraints, computational resource constraints, radio resource constraints, radio resource allocation over IoT edge constraints, latency constraints, and task execution constraints. It is hence formulated as follows:

(1) $$\begin{array}{c} \underset{a,\theta ,f}{\min}\sum_{i=1}^{N}a\left(i\right)\left(e_{c}\left(i\right)\right)+C\left(i\right)\left(1-k\left(f^{2}\left(i\right)\right)a\left(i\right)\right),\\ C_{1}:\sum_{i=1}^{N}f\left(i\right)\leq F,\\ C_{2}:0\leq f_{i}\leq a_{i}*F,\\ C_{3}:\sum_{i=1}^{N}\theta_{i}\leq L,\\ C_{4}:0\leq \theta_{i}\leq a_{i}L,\\ C_{5}:a_{i}\in \left\{0,1\right\},\\ C_{6}:\frac{C\left(i\right)}{f\left(i\right)}\left(1-a\left(i\right)\right)+a\left(i\right)\left(\frac{C\left(i\right)}{f\left(i\right)}+\frac{D\left(i\right)}{R\left(i\right)}\right)\leq T\left(i\right), \end{array}$$

where *α* is the execution vector, *θ* is the allocation of radio resource by 6G network, and *f* is the resource allocated in servers.

Furthermore, the tasks are executed locally while considering all the constrains *α*(*i*) = 0 [6], and the parameters are set as follows: *α*(*i*)*t*_*c*_(*i*) = 0 and *α*(*i*)*e*_*c*_(*i*) = 0 for local task execution.

- *C*1—resource allocation constraints
- *C*2—computational resource constraints
- *C*3—radio resource constraints
- *C*4—radio resource allocation over IoT edge constraints
- *C*5—latency constraint
- *C*6—task execution constraints

## 4. FNN Resource Allocation

A multinode FNN wireless healthcare model is often referred as the FNN wireless healthcare model that aims to improve the precision and performance and scales according to larger data size. The increasing size of input data learning for learning reduces significantly the training errors and enables error-free complex operations [8]. This allows the distributed FNN wireless healthcare model computing to draw significant decisions and conclusions over larger data sizes or in case of complex computing. The purpose-built distributed FNN wireless healthcare model operates in distributed edge computing environment that gains advantage in terms of its performance requirement, user cases, data size, and implementation effort.

The FNN wireless healthcare model learns the entire model with suitable parameters in the form of a matrix *W* ∈ *Rx* × *y* from the data stored across edge devices, where *x* and *y* represent the input and output dimensions. Consider a FL model at round *t* ≥ 0, where the server is allowed to distribute the current FL *W*(*t*) over the edge IoT devices. The edge devices update independently the FL model *W*(*t*) in terms of its local data. The data model after update is considered as *W*_1_(*t*), *W*_2_(*t*),…, *W*_*n*_(*t*), and hence, the update on the edge device say *i* is defined as *H*_*i*_(*t*) = *W*_*i*_(*t*) − *W*(*t*), where the edge devices *i* ∈ *S*(*t*). The edge device sends update to the edge node and then to the cloud centre, where it computes the global update based on the aggregation of edge device update.

(2) $$\begin{array}{c} W\left(t+1\right)\;=\;W\left(t\right)\;+\;H\left(t\right)\;\eta \left(t\right),\\ H\left(t\right)\;=n^{-1}{\left(t\right)}^{\sum_{i\in S\left(t\right)}H_{i}\left(t\right)}. \end{array}$$

The edge node is allowed to select *η*(*t*), the learning rate, and for faster computation, we have considered *η*(*t*) = 1. The FL is described for the DNN in next section, where it uses an individual matrix (*W*) in order of representing the parameters over each hidden layer. The parameters representing the full connected layers of the DNN in FL is hence described in the form of 2D matrix. On the other hand, the study aims to increase the efficiency of communication using the FNN wireless healthcare model that tends to reduce the communication and transmission cost of sending the updates *H*_*i*_(*t*) to the cloud centre. Whereas, the edge model considers learning the data from edge devices with constrained internet connectivity and its computational availability. To attain gradient computations, the loss function *L* with a parameter vector *w* is minimised using the learning problem to attain a closed form solution.

The study considers a simplest circulant matrix approach considering a vector *r* with viable error rates. Hence, the circulant matrix *R* ∈ *R*^*x*×*y*^ over a vector *r* is expressed as follows:

(3) $$\begin{array}{c} \text{Cir}\left(r\right)=R≔\left[\begin{array}{ccccc} r_{0} & r_{d-1} & \cdots & r_{2} & r_{1}\\ r_{1} & r_{0} & r_{d-1} & \cdots & r_{2}\\ \vdots & r_{1} & r_{0} & \cdots & \vdots \\ r_{d-2} & \vdots & \vdots & \ddots & r_{d-1}\\ r_{d-1} & r_{d-2} & \cdots & r_{1} & r_{0} \end{array}\right]. \end{array}$$

It has reduced the cost of storage to *O*(*d*) instead of *O*(*d*^2^). The computations using the circulant matrix uses fast Fourier transform to increase the speed of computations. Therefore, the computational complexity for a single-layered DNN (Figure 3) with a vector *r* having a dimension *d* is defined as *O*(*d*log*d*).

The modified circulant matrix *R* ∈ *R*^*d×n*^ is expressed as

(4) $$\begin{array}{c} R=SHG\Pi HB\text{,} \end{array}$$

where *G*, *S*, and *B* are the diagonal matrices, *H* is the Walsh–Hadamard matrix, and Π ∈ {0, 1}^*d*×*d*^ is the permutation matrix.

At the edge IoT device, the resource allocation should meet the user needs, and it should satisfy the QoS needs. Therefore, the set of resources in the edge node with the same service is stated as follows:

(5) $$\begin{array}{c} R\;=\;\left\{r_{1},r_{2},\ldots ,r_{n}\right\}. \end{array}$$

Considering all the attributes for resource allocation, the resource allocation is carried out based on user requirement, and the resource set *q*(*i*) is defined in terms of QoS attributes available for resource allocation.

(6) $$\begin{array}{c} q\left(i\right)=\left\{q_{1},q_{2},\ldots ,q_{n}\right\}, \end{array}$$

where *n* is the index resource with QoS attributes including response time, availability, cost, and reliability.

Here, the cost is estimated as follows:

(7) $$\begin{array}{c} p=UbD_{ed}\frac{\mu }{\varphi }, \end{array}$$

where *U* is the basic service cost, *µ* is the total requests, *φ* is the total service requests, *b* is the cost regulation, and *D*_*ed*_ is the edge IoT device.

If the resource is similar to the QoS attributes as demanded by edge device, the attributes set is thus expressed as follows:

(8) $$\begin{array}{c} u=\left\{u_{1},u_{2},\ldots ,u_{m}\right\}. \end{array}$$

The attribute matrix for QoS with respect to the resources is defined in the form of a decision matrix.

(9) $$\begin{array}{c} R={\left(r\left(ij\right)\right)}_{n\times m},\\ =\left(\begin{array}{cccc} r_{11} & r_{12} & \cdots & r_{1m}\\ r_{21} & r_{22} & \cdots & r_{2m}\\ \vdots & \vdots & \ddots & \vdots \\ r_{n1} & r_{n2} & \cdots & r_{nm} \end{array}\right), \end{array}$$

where *r*(*ij*) is the QoS attribute of *j*^th^ value over a resource (*i*).

The processing of the attribute matrix is considered meaningless if the units of measurement units are different for the QoS attributes. Hence, the relationship existing between user satisfaction and the QoS attributes is formulated as follows:

(10) $$\begin{array}{c} z\left(ij\right)=\left\{\begin{array}{cc} \frac{r\left(ij\right)-\min r\left(j\right)}{\max\;r\left(j\right)-\min\;r\left(j\right)}, & q>0,\\ \frac{\min\;r\left(j\right)-r\left(ij\right)}{\max\;r\left(j\right)-\min\;r\left(j\right)}, & q\leq 0. \end{array}\right. \end{array}$$

Here, an objective weight is set for each attribute, since the edge devices at the end-user have selected preference for a specific attribute that tends to affect the measurement directly, and it utilizes a weighted technique to estimate the preference.

(11) $$\begin{array}{c} d\left(u,i\right)=\sum_{j=1}^{m}\sqrt{w\left(j\right)*{\left(q\left(j\right)-u\left(j\right)\right)}^{2}},\\ \text{sim }d\left(u,i\right)=\frac{1}{1+d\left(u,i\right)}, \end{array}$$

where *w*(*j*) is the resource attribute weight, *d*(*u*, *i*) is the distance from ideal to edge node (*i*), and sim*d* (*u*, *i*) is the proximity degree [0, 1].

## 5. Performance Evaluation

In this section, the entire simulation is conducted in Matlab environment to study the effectiveness of the proposed model. This section focuses on the experimentation that has been conducted to verify the effectiveness of the FNN wireless healthcare model in helping resource allocation decisions regarding metrics like average success rate, job response time, and resource utilisation levels. Latency is calculated by finding the Euclidean distance between edge devices according to the distance model in [9]. Response time is a factor in resource allocation, and an edge device with a high-valued response time would be considered a failure-allocated task. The study uses three data centres with 100 servers, where each server consists of 6 cores with 5 hostings per server. The location of data centre is considered random with 30 ms response time and with 100 bytes low latency level.

FNN wireless healthcare model effectiveness is studied through 3 different performance metrics in this study. For the first time, the average response time of each allocated resource to the edge device is measured when computing the impact of cloud servers on the network node. Also, the average task utilisation is estimated at the node where the task is created, and third, the likelihood of tasks allocated per failure is calculated. Each of these 3 responses is analysed under consideration of response time constraints, and eventually, network throughput is estimated.

### 5.1. Influence of Data Centre with Core Server

According to estimations, the performance of three techniques on three different servers connected to a data centre is expected. This study will lead to the increase of between 200 and 2000 cloud servers. Careful consideration has been given to the servers, such that the total servers that are connected to the cloud data centre have the same number of servers as those connected to a microdata centre.  Figure 4(a) shows the total servers connected to edge servers for each allocated task. The FNN wireless healthcare model improves the performance relative to the current FL and DNN when more resources are shared among the edge nodes. There is an optimum level of performance even if only a small number of servers are connected to the edge servers.

In Figure 4(b), higher-order use of resources is illustrated. One microdata centre of edge handles over 150 cloud servers, allowing for greater overall resource utilisation than just the amount of time spent on scare resources. Additionally, as more servers are added, the resource utilisation success rate increases and never reaches 99.99%. The higher the burden, the less successful the existing FL and DNN methods are. As these methods have a harder time handling the increased burden, they have a negative impact on the success rate. However, missing the response time constraint (Figure 4(c)) is a significant barrier to making neighbourhood edge data centres a reality. Constrained response time, limited resource utilisation, and improved success rate were found to improve overall performance with the experimental results.

### 5.2. Influence of Data Centre on the Entire Network

This proposed study confirms that the FNN wireless healthcare model achieves the desired performance even when run on several edge nodes or in microdata centres. Here, we go from a state with around 200 edge nodes to around 20 edge nodes, and then, groups of 20 edge nodes are grouped together with each group assigned to a service provider.  Figure 3(a) shows that as edge nodes increase, response time decreases from 20 to 10 ms. It is because the edge nodes and edge devices are farther apart today. Another feature that already exists functions with a similar range; response time grows from 18 ms to 21 ms. Since the cloud centre appears unaffected by available edge nodes, it can be concluded that the cloud centre does not rely on the availability of nodes on the edge. Figures 3(b) and 3(c) illustrate an increase in the amount of resources used by the FNN wireless healthcare model compared to the existing FL and DNN. Additionally, the proposed mechanism has a higher success rate than in Figure 3(c). The findings demonstrate that the FL and DNN are better than other systems at significantly increasing performance.

### 5.3. Impact of Response Time Constraint

The average response time tends to increase as the response time constraint increases (Figure 5(a)). This increases scalability, as the workloads can be distributed fairly between edge devices and edge nodes. Because of their distance, their response time tends to be impacted. For example, in Figure 5(b), the resource utilisation is compared, and it is found that the increased response time constraint causes the utilisation to increase. Performance similar to the FNN wireless healthcare model can be achieved if the response time constraint at the edge nodes is increased. The edge node can provide a higher percentage of completed tasks in cloud locations because it has a lower response time constraint. Furthermore, as shown in Figure 5(c), the average success rate increases when reresponse time constraints are extended. When compared to other existing resource allocation methods, the proposed solution obtained an average success rate of 99.9%. According to the results, the FNN wireless healthcare model has an edge over other methods, even when response time limits are present.

## 6. Conclusion

In this study, the FNN wireless healthcare model applies its distributed resource allocation settings to allocate optimal resources to the edge devices. To support the distributed settings of edge intelligence, FL adjustments are implemented. In terms of improved average success rate, higher resource utilisation, and increased network throughput, the design of computational and storage cost reduction in the edge network and in hidden layers has been a big success. Conventional methods demonstrate higher scalability in distributed deep learning models compared to the FNN wireless healthcare model. In future, metaheuristic models can be deployed to create shear intelligence on detecting optimal resource allocation to edge devices.

## Figures and Tables

**Figure 1:** 6G edge computing framework.

**Figure 2:** The service request in cybertwin for resource allocation.

**Figure 3:** (a) Response time w.r.t the influence of data centre. (b) Resource utilisation w.r.t the influence of data centre. (c) Success rate w.r.t the influence of data centre.

**Figure 4:** (a) Response time w.r.t the influence of connected data centre. (b) Resource utilisation w.r.t the influence of connected data centre. (c) Success rate w.r.t the influence of connected data centre.

**Figure 5:** (a) Response time w.r.t response time constraints. (b) Resource utilisation w.r.t response time constraints. (c) Success rate w.r.t response time constraints.

## Data Availability

The datasets used and/or analysed during the current study are available from the corresponding author upon request.

## References

[1] Weisong S., Hui S., Jie C., Quan Z., Wei L. (2017). Edge computing—an emerging computing model for the Internet of everything era. *Journal of Computer Research and Development*.

[2] Yu Q., Ren J., Fu Y., Li Y., Zhang W. (2019). Cybertwin: an origin of next generation network architecture. *IEEE Wireless Communications*.

[3] Nayak S., Patgiri R. (2021). 6G communication technology: a vision on intelligent healthcare. *Health Informatics: A Computational Perspective in Healthcare*.

[4] Kaiser M. S., Zenia N., Tabassum F. 6G access network for intelligent internet of healthcare things: opportunity, challenges, and research directions.

[5] Shi W., Cao J., Zhang Q., Li Y., Xu L. (2016). Edge computing: vision and challenges. *IEEE Internet of Things Journal*.

[6] Guan Y., Lu R., Zheng Y., Zhang S., Shao J., Wei G. (2021). Toward privacy-preserving cybertwin-based spatio-temporal keyword query for ITS in 6G era. *IEEE Internet of Things Journal*.

[7] Yan S., Ye Q., Zhuang W. (2021). Learning-based transmission protocol customization for VoD streaming in cybertwin-enabled next generation core networks. *IEEE Internet of Things Journal*.

[8] Halevy A., Norvig P., Pereira F. (2009). The unreasonable effectiveness of data. *IEEE Intelligent Systems*.

[9] Goonatilake R., Bachnak R. A. (2012). Modeling latency in a network distribution. *Network and Communication Technologies*.

[10] Adhikari M., Munusamy A., Kumar N., Srirama S. N. (2021). Cybertwin-driven resource provisioning for IoE applications at 6G-enabled edge networks. *IEEE Transactions on Industrial Informatics*.

[11] Wang Y., Sheng M., Wang X., Wang L., Li J. (2016). Mobile-edge computing: partial computation offloading using dynamic voltage scaling. *IEEE Transactions on Communications*.

[12] Rodrigues T. K., Liu J., Kato N. (2021). Application of cybertwin for offloading in mobile multi-access edge computing for 6G networks. *IEEE Internet of Things Journal*.

[13] Liang H., Li H., Zhang W. (2021). A combinatorial auction resource trading mechanism for cybertwin based 6G network. *IEEE Internet of Things Journal*.

[14] Juneja S., Gahlan M., Dhiman G., Kautish S. (2021). Futuristic cyber-twin architecture for 6g technology to support internet of everything. *Scientific Programming*.

[15] Wang S., Tuor T., Salonidis T. (2019). Adaptive federated learning in resource constrained edge computing systems. *IEEE Journal on Selected Areas in Communications*.

[16] Yang Q., Liu Y., Chen T., Tong Y. (2019). Federated machine learning. *ACM Transactions on Intelligent Systems and Technology*.

